# Prediction Model of Adverse Effects on Liver Functions of COVID-19 ICU Patients

**DOI:** 10.1155/2022/4584965

**Published:** 2022-04-25

**Authors:** Aisha Mashraqi, Hanan Halawani, Turki Alelyani, Mutaib Mashraqi, Mohammed Makkawi, Sultan Alasmari, Asadullah Shaikh, Ahmad Alshehri

**Affiliations:** ^1^College of Computer Science and Information Systems, Najran University, Najran, Saudi Arabia; ^2^Department of Clinical Laboratory Sciences, College of Applied Medical Sciences, Najran University, Najran, Saudi Arabia; ^3^Faculty of Applied Medical Sciences, King Khalid University, Abha, Saudi Arabia

## Abstract

SARS-CoV-2 is a recently discovered virus that poses an urgent threat to global health. The disease caused by this virus is termed COVID-19. Death tolls in different countries remain to rise, leading to continuous social distancing and lockdowns. Patients of different ages are susceptible to severe disease, in particular those who have been admitted to an ICU. Machine learning (ML) predictive models based on medical data patterns are an emerging topic in areas such as the prediction of liver diseases. Prediction models that combine several variables or features to estimate the risk of people being infected or experiencing a poor outcome from infection could assist medical staff in the treatment of patients, especially those that develop organ failure such as that of the liver. In this paper, we propose a model called the detecting model for liver damage (DMLD) that predicts the risk of liver damage in COVID-19 ICU patients. The DMLD model applies machine learning algorithms in order to assess the risk of liver failure based on patient data. To assess the DMLD model, collected data were preprocessed and used as input for several classifiers. SVM, decision tree (DT), Naïve Bayes (NB), KNN, and ANN classifiers were tested for performance. SVM and DT performed the best in terms of predicting illness severity based on laboratory testing.

## 1. Introduction

The COVID-19 pandemic was declared a health emergency in 2020. Many people have died during the pandemic, particularly in the early stages, due to a lack of understanding of the virus. COVID-19 has led to over 3.5 million deaths worldwide [1–3]. Patients infected with COVID-19 may experience no symptoms or severe illness that can lead to death [4]. The virus continues to evolve, with concerning mutants emerging all over the world [5]. This is an alarming situation and requires a better understanding of the disease in order to save more lives. Critical cases of COVID-19 could result in organ failure and death. Lung failure is the most common complication, but other organs can also be affected by the virus. In fact, multiorgan failure involving the lungs, kidneys, liver, cardiovascular system, and gastrointestinal tract (GIT) can also occur [6]. Additionally, people who already suffer from liver diseases, such as cirrhosis, are at a higher risk of decompensation and death during COVID-19 infection [7]. Organ failure is serious; therefore, managing infection is of interest.

The liver is a vital organ, and its failure could be fatal. COVID-19 patients can have mild to severe symptoms and may develop acute hepatic failure [6]. According to the proposed mechanism, hepatic failure occurs due to multiple factors. These include angiotensin-converting enzyme 2 (ACE2), a SARS-CoV-2 receptor found in multiple organs including the liver, and cytokine storm, which occurs as a result of inflammatory mediators, endothelial dysfunction, coagulation abnormalities, and inflammatory cell infiltration into the organs [6]. Direct cytotoxicity caused by active virus replication in the liver could result in liver cell damage. Furthermore, hypoxic liver damage is exacerbated by severe lung failure and disease. Cardiac congestion as a result of SARS-CoV-2 disease-induced right-sided heart failure can also result in liver damage. Furthermore, people with preexisting liver disease, as well as drug-induced liver injury, experience exacerbation [8]. To avoid COVID-19 disease complications, it is critical to detect liver damage early and understand its extent.

The exact molecular mechanism of the above-mentioned hepatic injury is unknown. However, SARS-CoV-2 viral RNA has been detected in liver tissue using qRT-PCR, indicating that the virus can affect liver cells [9]. It is still unclear where virus replication occurs in the liver, but an intact virus was found in the cytoplasm of COVID-19 patients with abnormal liver function tests [10]. Viral receptors have been found on the surface of host cells, which could explain the viral tropism towards the specific tissue. SARS-CoV-2 enters the cell via the virus's S protein, which binds to host cell receptors such as ACE2 and TMPRSS2 [11]. The expression of ACE2 and TMPRSS2 receptors is low but still presents in the hepatic cells [12]. Moreover, it is a noteworthy finding that the expression of ACE2 receptors is increased in both humans and mice with liver fibrosis [13]. Interestingly, hypoxic cases were found to be associated with increased expression of ACE2 receptors, which could explain the mechanism of ACE2 receptor upregulation in COVID-19 patients due to lung damage [13].

A variety of factors in SARS-CoV-2 infection can result in hypoxia-induced liver damage. Heart failure, lung failure, and sepsis are the three most serious of these. These factors account for 90% of all cases of hypoxic damage in COVID-19 cases. Moreover, right-sided heart failure causes liver congestion due to raised central venous pressure (CVP). Hypoxia and liver congestion cause centrilobular necrosis over time [14]. Many known hepatotoxic agents have been used to treat COVID-19 disease. These drugs include corticosteroids and antivirals. Corticosteroids have been found to cause steatosis, and hepatotoxicity is caused by antivirals such as ritonavir and remdesivir [8].

Liver enzymes, which were found to be elevated in a number of COVID-19 cases, can be used to detect liver damage. Although the incidence of liver involvement has been reported in several COVID-19 cases, the extent of the prevalence of hepatic damage remains unknown [15]. Elevated liver enzymes, particularly alanine aminotransferase (ALT) and aspartate aminotransferase (AST), have been reported in 14% to 53% of patients [16]. There is a strong correlation between the severity of the disease and the extent of liver involvement [16]. According to research, mild COVID-19 disease causes a mild elevation of liver enzymes, whereas severe disease causes a significantly higher level of liver enzymes [16, 17]. In a study of 222 COVID-19 patients, 28.2% had elevated liver enzymes. The reason for this elevation, however, was not specified, and it could have been preexisting [18]. Furthermore, a study of 417 COVID-19 patients discovered that 76.3% of the total sample had abnormal liver function tests. During their hospital stay, 21.5% suffered a liver injury. Their levels of liver enzymes significantly increased within two weeks of hospitalization. According to the findings of the study, patients with significantly elevated liver enzymes are at a higher risk of developing severe disease [19, 20].

Machine learning (ML) is being introduced to medicine and used as artificial intelligence (AI) to create predictive models based on data patterns. Machine learning can also be used to create a predictive model of liver involvement [21]. Machine learning (ML) is currently being used to predict the possibility of fatty liver disease [22], the success of liver transplants [23], and other hepatic conditions. However, there is still no firm agreement on which machine learning algorithm is best to use as an illness-prediction method. The outcome of patients with raised liver enzymes admitted to the ICU with COVID-19 disease should be predicted using machine learning (ML), which could be useful in disease management.

Millions of people have died as a result of the SARS-CoV-2 virus, and more people are becoming infected every day. Elevated liver enzymes are linked to the severity of the illness, which can be fatal. Early detection of disease warning signs, on the other hand, can be beneficial. During COVID-19 disease, elevated liver enzymes are seen, and their level is related to the severity of the disease and the extent of liver damage. Therefore, monitoring of liver enzymes in ICU SARS-CoV-2 patients can be used to improve their health. Moreover, with the progress of machine learning toward improved screening methods for the severity of COVID-19 infection, the numbers of infected individuals have decreased significantly, motivating artificial intelligence (AI) scientists and medical physicians to employ this subject more thoroughly in the health sector. Algorithms in machine learning are developed to allow computers to learn. ML algorithms can be used for classification problems, which have been applied in the medical field to help in the early diagnosis of several diseases. However, there are specific difficulties with these computational methods, including the feature-selection step in prediction models. Other studies have used a different methodology for feature selection, such as a pivot table in [24] and a P-value in [25].

In this paper, we propose a model to predict liver damage based on data patterns using supervised learning techniques. The model is named detecting model for liver damage (DMLD), and it employs machine learning algorithms to assist in the early detection of the risk of liver damage. It will support healthcare professionals to diagnose the disease at its early stages. Data from blood tests of COVID-19 patients admitted to the ICU were collected, cleaned, and prepared to be used as input for the model. Secondly, we designed the DMLD model that prepares the data set in the preprocessing phase by addressing the missing values and applying the normalization approach. Then, the DMLD model identifies the most relevant features in the feature-selection phase by applying a filtering method. Consequently, five machine learning classifiers were examined in order to find the best-performing algorithms; which are support vector machine (SVM), decision tree, Naïve Bayes (NB), K-nearest neighbors (KNN), and artificial neural network (ANN). These methods have certain drawbacks; for example, NB is simple and suitable for large data sets. However, it assumes that numeric properties have a normal distribution. Data preparation is easier with the DT but is dependent on the sequence of the characteristics. KNN, SVM, and ANN are computationally expensive [26]. In our study, the performance of the DMLD model was evaluated on the collected data set, and the results show that the accuracy, precision, and recall of the SVM and DT classifiers are better than others. Therefore, we considered SVM and DT the likely best algorithms for detecting the risk of liver damage.  Figure 1 illustrates the study framework.

The rest of the paper is structured as follows. First, we present the related work. Then, we explain the DMLD prediction model in detail, describing the data set details and the DMLD stages with the classification algorithms. Then, we present the results and discuss the performance of the DMLD model, including the measurement of classification techniques. Finally, we provide the conclusions and identify the future directions.

## 2. Related Work

Machine learning approaches have attracted the attention of many researchers and have been applied in different disciplines such as medicine, the economy, and education. Moreover, machine learning plays an essential role in the medical field, contributing to various health sectors such as the early diagnosis of disease and treatment. Liver disease is a common health issue. Therefore, early diagnosis of the risk factors will help medical physicians predict the development of the disease [27].

Ayeldeen et al. [28] highlighted that the positive prediction of different stages of liver fibrosis can be predicted by biochemical markers. The decision tree algorithm has been considered to predict the risk of liver fibrosis, and the model has been tested using a data set that includes laboratory tests and fibrosis markers. Another study [29] compared the performance of different algorithms (logistic regression, KNN, ANN, and SVM) to assess liver disease detection. Additionally, Sontakke et al. [30] utilized backpropagation and SVM algorithms to predict liver disease. Thirunavukkarasu et al. [24] applied logistic regression, SVM, and KNN for predicting liver disease based on the evaluation of accuracy, sensitivity, and specificity (recall). Moreover, Venkata Ramana et al. [31] studied the performance of various machine learning algorithms using different metrics (accuracy, precision, sensitivity, and specificity).

A support vector machine (SVM) is considered a promising machine learning algorithm for classification problems. In addition, there are many studies that apply the SVM algorithm to text classification, face recognition, and bioinformatics. The performance of the SVM algorithm is often good compared to other techniques [32–34]. Another machine learning algorithm is the Naïve Bayes classifier, which is a simple probabilistic classifier applying Bayes' theorem. In addition, the Naïve Bayes classifier estimates the means and variances of the variables for classification using a small amount of training data [35]. Moreover, decision tree (DT) and K-nearest neighbors (KNN) are supervised learning algorithms considered suitable for addressing both classification and regression problems [36–38]. Another popular machine learning method is the artificial neural networks (ANN) that are inspired by the neural networks of the human brain [39].

Deep learning has exploded significantly in scientific computing, with its techniques being utilized by a variety of fields to solve complicated problems. To perform certain tasks, all deep learning algorithms employ various forms of neural networks. Neural networks are used in deep learning to perform complex computations on massive amounts of data. It is a form of machine learning that is based on the human brain's structure and function. The performance of classification is improved the most when the machine learning algorithm is updated with a deep learning algorithm. Over the last few years, there has been a lot of development in the use of neural networks for feature extraction in object identification problems. For example, Zhang et al. created Deep-IRTarget, a unique backbone network composed of a frequency feature extractor, a spatial feature extractor, and a dual-domain feature resource allocation model, to cope with challenges in feature extraction [40]. Moreover, the deep learning algorithm is employed in burnt area mapping with the use of Sentinel-12 data [41]. Zhang et al. present a Siamese self-attention (SSA) classification approach for multisensor burnt area mapping, and a multisource data set is created at the object level for training and testing. Zhang et al. implement a robust, multicamera, multiplayer tracking framework. They used a deep learning algorithm in their system to understand the impact of player identification and the most distinguishing data [42]. Furthermore, deep learning algorithms have been used to identify COVID-19 using X-ray processing. For example, several studies [43–45] present a rapid, robust, and practical method for detecting COVID-19 from chest X-ray images. According to experiments by Mahajan et al. [43], DenseNet is the best classifier to utilize as a base network with SSD512, especially for the problem of identifying COVID-19 infection in chest X-ray images. Mahajan et al. [44] developed a model for detecting COVID-19 from chest X-ray images. They used ResNet101 as the basic network and implemented transposed convolution, prediction modules, and information injection into the DSSD network. The artificial intelligence-based detection models can significantly contribute to the attainment of massive and high-performing screening programs in various medical sectors.

## 3. Proposed Method

The main contribution of this study is the design of a prediction model to detect the risk of liver damage, called the detecting model for liver damage (DMLD).

### 3.1. Detecting Model for Liver Damage (DMLD)

In this study, we design a prediction model for adverse effects on liver functionality of COVID-19 ICU patients called detecting model for liver damage (DMLD). The methodology of this study involves five stages, which are data collection, data preprocessing, feature selection, classifiers, and evaluation and then result collection.  Figure 2 illustrates the system architecture of the DMLD prediction model. Moreover, a detailed explanation of the DMLD model will be presented in the following subsections.

#### 3.1.1. Material

The data set used in this research was obtained from two main hospitals in the southern region of Saudi Arabia (Asir Central Hospital (ACH) in Asir and King Khalid Hospital in Najran). A total of 140 patients were included in the data set. The study was limited to patients with positive COVID-19 infection who were admitted to the intensive care unit (ICU). Ethical approval (REC No.: REC-11-1O-2020) for this study was obtained from the Regional Committee for Research Ethics, Directorate of Health Affairs, Asir Region, Ministry of Health, Saudi Arabia, and ethical approval (IRB Log Number: 2020-24E) for this study was obtained from the Regional Committee for Research Ethics, Directorate of Health Affairs Najran, Ministry of Health, Saudi Arabia.

The data set has recent laboratory results and missing values are very minimal. The laboratory results contain 20 numeric attributes as follows: creatinine, glucose, sodium, potassium, calcium, phosphorus, magnesium, chloride, uric acid, urea, total protein, TG, AST, ALT, cholesterol-VLDL, cholesterol-LDL, cholesterol-HDL, and LDH. The class presented in this data set is binary, which refers to whether a patient has damage in the liver functionality or not based on abnormal liver enzymes. Prediction of liver damage is very likely based on elevated liver enzymes, which are released from the liver as a result of liver injury. SARS-CoV-2 has been reported to cause infection of the liver via binding to angiotensin-converting enzyme 2 (ACE2) on cholangiocytes, which are a population of liver cells [46]. The binding of SARS-CoV-2 to ACE2 will facilitate viral entry into the liver, causing damage to liver cells (hepatocytes) [46, 47]. Levels of ALT and AST in our data, which are specific liver enzymes, were significantly increased indicating liver injury. We identified liver damage based on normal values of liver enzymes.  Table 1 shows the liver enzymes along with their normal and disturbing values. Any patient with increased liver enzymes levels is considered at risk of liver damage. In the study data set, the percentage of possible liver damage is 50%.  Table 2 shows the data set attributes and the obtained results from the laboratory, which were used to examine the DMLD prediction model.

#### 3.1.2. Data Preprocessing

The aim of the data preprocessing phase is to clean the data set in order to use it as input for classifier algorithms and then to provide more accurate observation. One of the significant issues in the collected real data is missing values. These missing values are very rare, at 4%; therefore, they were excluded from the data set. Another important aspect of data preprocessing is normalization, in which all attributes should have equal weight. In a simple ward, a common scale or range can be used. A popular and widely used normalization technique is min-max normalization, which is applied in this study. The min-max normalization technique transforms and rescales the data between the range [0, 1] by the following equation:

(1) $$\begin{array}{c} x^{\prime }=\frac{x-\min_{F}}{\max_{F}-\min_{F}}, \end{array}$$

where min_*F*_ and max_*F*_ are the minimum and the maximum values of the feature *F*, respectively. The original and the normalized value of the attributes, *F*, are represented by *x* and *x*′, respectively [48].

#### 3.1.3. Features Selection

The data collected from the blood test will have plenty of different features with different information. Therefore, the feature-selection step is applied to reduce the number of relevant features in the data set, and consequently, the size of the problem will be reduced, and we can obtain a better prediction for the risk of liver damage. In this research, the filter method has been followed in order to rank the importance of *k* features in the data set based on the relationship between the features and the target variable [49]. In addition, the correlation between the selected features was examined in order to understand the data set and the relationship between the features.

#### 3.1.4. Classifiers

In the DMLD model, five machine learning classifiers have been used, which are support vector machine (SVM), decision tree (DT), Naïve Bayes (NB), K-nearest neighbors (KNN), and artificial neural network (ANN). These classifiers were used to determine the risk of liver damage and the selection of these classifiers is based on the following characteristics.

Support vector machine (SVM): Support vector machines (SVM) are extensively used in medical applications. The SVM algorithm with class labels of unknown data is used to develop an effective model for predicting disease. SVM is used [50] in both classification and regression [51]. The data points in the SVM model are represented in space and divided into groups, with all points with comparable qualities falling into the same group. The given data set is treated as a *p*-dimensional vector in linear SVM, which can be split by a maximum of *p*-1 planes termed hyperplanes. As shown in Figure 3, these planes divide the data space or define the boundaries between data groups for classification or regression issues. On the basis of the distance between the two classes it separates, the optimal hyperplane can be chosen among a large number of hyperplanes. The maximum-margin hyperplane is the plane with the largest margin between the two classes [52, 53]. For *n* data points, the formula is
  (2) $$\begin{array}{c} \left(\overset{⟶}{x_{1}},y_{1}\right),\ldots ,\left(\overset{⟶}{x_{n}},y_{n}\right), \end{array}$$
where *x*_1_ is a real vector and *y*_1_ is the class to which *x*_1_ belongs and is either 1 or −1. The distance between the two classes *y*=1 and *y*=−1 can be maximized by constructing a hyperplane, which is defined as follows:
  (3) $$\begin{array}{c} \overset{⟶}{w}\cdot \overset{⟶}{x}-b=0, \end{array}$$
where $\overset{⟶}{w}$ is the normal vector and $b/\left\|\overset{⟶}{w}\right\|$ is the hyperplane's offset along $\overset{⟶}{w}$.
In an SVM model, tuning parameters help optimize the classification results based on the specific data points provided [54]. One of them may be the kernel, a mathematical function that accepts data as input and transforms it into the required format. These functions return the inner combination between two points in a sufficient space, which might be linear, nonlinear, radial base function (RBF), polynomial, or sigmoid.
Decision Tree (DT): The decision tree classifier is considered a supervised learning algorithm [36]. Compared with other supervised learning algorithms, a decision tree algorithm can be used for dealing with both classification and regression problems. The overall perspective of using a DT is to create a preparation model that can predict class or assessment of target factors by taking decision standards derived from training data. The decision tree classifier can be a fast learner when constructing a decision/regression tree utilizing acquired information as the splitting criterion, and it prunes the tree by minimizing error pruning [37].
Naïve Bayes (NB): A Naïve Bayes classifier is a classical probabilistic classifier dependent on performing Bayes' theorem within a highly independent assumption [35]. The fundamental probability model would be as descriptive as the self-determining feature model. The basic assumption in the Naïve Bayes classifier is that the presence of a specific feature of a class is unassociated with the presence of other features [55]. Even if the assumption is not accurate, the Naïve Bayes classifier performs reasonably well. The Naïve Bayes classifier has another advantage, which is that it only requires a small data set for the training stage in order to compute the means and variances of the essential variables for classification. For each label, only the variances of the variables need to be computed, not the whole covariance matrix, because unassociated variables are unspecified. The kernel of the Naïve Bayes operator can be formulated on numerical attributes. This is clearly achieved by applying Bayes' theorem and kernel density estimation.
  (4) $$\begin{array}{c} \hat{P}\left(y=j|x_{0}\right)=\frac{{\hat{\pi }}_{j}{\hat{f}}_{j}\left(x_{0}\right)}{\sum_{k=1}^{k}{\hat{\pi }}_{k}{\hat{f}}_{k}\left(x_{0}\right)}, \end{array}$$
where $\hat{\pi }$ is an estimate of the prior probability of class *j*, and normally, $\hat{\pi }$ is the sample proportion falling into the *j*^th^ classification. ${\hat{f}}_{j}$ is the predictable density at *x*_0_ depending on a kernel density fit, including only perceptions from the *j*^th^ class. This is essentially similar to discriminant analysis, only instead of assuming normality, it estimates the probability density of the classes utilizing a nonparametric method, Patrick.
K-Nearest Neighbors (KNN): In machine learning, KNN is one of the most fundamental classification algorithms, and it produces excellent results [36]. KNN is a nonparametric, instance-based learning algorithm and can be used to solve problems involving classification and regression. In classification, KNN is used to determine which class a new unlabeled item belongs to. In any case, the KNN makes a shot at the assumption that comparable samples are close fits [38]. KNN sorts a sample into the most decided class among K neighbors. K is usually odd and is restricted by how the classification algorithms can be adjusted [56]. This will be achieved by computing the distance between the data points that are nearest to the samples by using methods such as Euclidean distance, Manhattan distance, Hamming distance, or Minkowski distance. In this study, the Euclidean distance metric was used in the final model for calculating the distance between data points. Following the calculation of the distance, the K closest neighbors are chosen, and the resultant class of the new object is determined using the votes of the neighbors [51, 57].
Artificial neural network (ANN): The functionality of an artificial neural network (ANN) is similar to that of the human brain [39]. It resembles a network of nodes known as artificial neurons. All of these nodes communicate with each other to transmit information. The neurons in the ANN can be represented by a state (0 or 1), and each node might have a weight attached to it that determines its relevance or strength in the system. The ANN structure is separated into layers with many nodes; data flow from the first layer (input layer) to the output layer after passing through intermediary levels (hidden layers). Every layer turns the data into relevant information before delivering the target output [58]. The processes of transfer and activation are crucial in the functioning of neurons. The sum of all the weighted inputs is calculated using the transfer function:

(5) $$\begin{array}{c} z=\sum_{x=1}^{n}w_{i}x_{i}+w_{b}b, \end{array}$$

where *b* is the bias value, which in most cases is 1. Furthermore, the activation function essentially flattens the transfer function's output into a specified range. The activation function could be linear or nonlinear and can be expressed simply as follows:

(6) $$\begin{array}{c} f\left(z\right)=z, \end{array}$$

Since no data restrictions are provided by the activation function, the sigmoid function is employed [51], which is written as follows:

(7) $$\begin{array}{c} a=\sigma \left(z\right)=\frac{1}{1+e^{-z}}. \end{array}$$

#### 3.1.5. Evaluation

The proposed model's (DMLD) performance was evaluated using the measurement performance of several classification algorithms. Various evaluation methodologies, such as accuracy, precision, and recall, are used. The following is a list of their definition.

Accuracy: The percentage of accurate and valid classifications is known as the accuracy [59]. To calculate the accuracy, the true positive (TP), false positive (FP), true negative (TN), and false negative (FN) values are required.

(8) $$\begin{array}{c} \text{Accuracy}=\frac{\text{TP}+\text{TN}}{\text{TP}+\text{FP}+\text{TN}+\text{FN}}. \end{array}$$

Precision: Positive predictive value is another term for precision. It shows the percentage of positive outcomes successfully predicted by classifier algorithms.

(9) $$\begin{array}{c} \text{Precision}=\frac{\text{TP}}{\text{FP}+\text{TN}}. \end{array}$$

Recall: Recall is also referred to as sensitivity or true positive rate because it mostly displays the method's positive outcomes [60]. The affectability evaluation determines the patient's ability to be identified by their liver condition.

(10) $$\begin{array}{c} \text{Recall}=\frac{\text{TP}}{\text{TP}+\text{FN}}, \end{array}$$

The evaluation variables that are used in the performance measurement, which is the confusion matrix, are determined as follows. True positive (TP): The outcome of the prediction properly identifies the presence of the risk of liver damage in a patient. False positive (FP): The outcome of the prediction mistakenly identifies a patient as having the risk of liver damage. True negative (TN): The outcome of the prediction properly rejects the possibility of a patient being at risk of liver damage. False negative (FN): The outcome of the prediction mistakenly rejects the possibility of a patient being at risk of liver damage.

Tenfold cross-validation is used to avoid the problems of over- and underfitting [61]. Then, the previous measurement performance is used to evaluate the classification systems' performance. Accuracy reflects how accurate our classifier is in determining whether or not a patient is at risk of liver damage. Precision also has been applied to measure the classifier's ability to make an accurate, positive prediction of the risk of liver damage. Additionally, sensitivity or recall is employed in our research to determine the percentage of actual positive cases of risk of liver damage that the classifier properly detects.

## 4. Results and Discussion

In this study, the DMLD model is proposed to contribute to the prediction of the risk of liver damage using laboratory blood tests. The DMLD model was implemented and examined in the Python 3.8 programming language via Anaconda Navigator [62]. In addition, different measurement metrics (accuracy, precision, and recall) were considered to assess the performance of the DMLD model. This was conducted using different machine learning classifiers to predict the risk of liver damage. Tenfold cross-validation was considered in order to validate the results. The data set in this study includes 140 COVID-19 ICU patients with 20 features, as shown in Table 1. Normalization is used for scaling the data because the data set variables (e.g., ALT, AST, and LDH) have different ranges of values. For example, LDH for a single patient is 499 U/L, and ALT and AST are 90 U/L and 34 U/L, respectively. Therefore, we applied different normalization algorithms such as min-max and mean, but the results did not show any difference. After applying the feature-selection step in the DMLD model, the results revealed that the three highest-scoring features were AST, ALT, and LDH, as shown in Figure 4. These selected features agreed with clinically reported features related to liver injury. ALT and AST are specific liver enzymes, and hence, they are considered markers for liver injury and failure [63, 64]. Moreover, increased LDH levels have been reported in patients with acute liver failure [65, 66]. Correlation coefficients of selected features were applied to screen for possible correlation. The linear relationship among selected features was defined as follows: positive correlation for *r* = 0.01 to 1.0 (where 1.0 was considered strong). As illustrated in Figure 5, a heat map was used to present our results, in which ALT and AST showed a significant positive correlation with *r* = 0.96. This correlation between ALT and AST is not surprising, since they are already approved scientifically as liver function markers. However, in agreement with our selection of LDH as an important feature, the heat map results interestingly revealed a very strong correlation between LDH and both specific liver enzymes ALT and AST, with *r* = 0.94 and *r* = 0.97, respectively.

Figure 6 describes the performance of the different classifiers used in the DMLD model, which are support vector machine (SVM), DT, Naïve Bayes (NB), K-nearest neighbors (KNN), and artificial neural network (ANN). In the validation phase, the model was tested in two different methods, namely train-test split and tenfold cross-validation. In the train-test split approach, the data set was divided into two parts, training and testing. The DMLD model was trained with 80% of the data set, and the remaining data were used for testing the DMLD model, by which preliminary results were gained. In addition, the tenfold cross-validation was applied in order to avoid overfitting, as shown in Table 3 and Figure 6.

Table 3 and Figure 6 show that the accuracy of SVM is 0.87 and that of DT is 0.85, while for the Naïve Bayes, KNN, and ANN, it is 0.71. Therefore, SVM and DT achieved higher accuracy than other classifiers (Naïve Bayes, KNN, and ANN). In addition, we tried to study the impact of different layers on the ANN performance by measuring the accuracy of the ANN algorithm, but the results showed no effect on the algorithm performance, as presented in Table 4. Regarding precision, SVM achieved the highest score, with 0.95, and the score was 0.93 for DT. For Naïve Bayes, KNN, and ANN classifiers, the precision values were found to be 0.5, 0.5, and 0.49, respectively. The recall score of SVM was the highest, at 0.95, and this score was 0.93 for DT. For Naïve Bayes, KNN, and ANN classifiers, recall scores were 0.5, 0.5, and 0.49, respectively.

The performances of five classifiers in the DMLD model have been examined. Therefore, from the above results, it can be noted that SVM and DT are the most sufficient classifiers in the DMLD model for predicting the risk of liver damage in COVID-19 patients. In agreement with our study, performances of the SVM [30] and DT [28] algorithms have been utilized to predict liver disease. SVM has shown the best performance. This is perhaps due to its ability to classify classes and generate a hyperplane that segregates classes after data transformation. Therefore, early diagnosis of risk factors by machine learning models such as SVM could assist in planning medical decisions and treatment.

## 5. Conclusions and Future Work

The effects of COVID-19 on the body are widespread. The early diagnosis of liver damage due to COVID-19 can contribute to making medical decisions. Therefore, this study suggests that the DMLD model can help in the prediction of the risk of liver damage during SARS-CoV-2 infection. To evaluate the DMLD model, data on COVID-19 and ICU patients were collected, preprocessed, and then used as an input for different classifiers. The performances of SVM, DT, Naïve Bayes, KNN, and ANN classifiers were evaluated. SVM and DT showed the best performance for predicting the diagnosis of disease severity based on laboratory tests. Therefore, this model could be applied for the prediction of other diseases. The further study of our work can be considered from two directions. Firstly, the prediction of different risk levels of liver diseases could be extended, as the current work is limited to the DMLD model. Secondly, our data were limited to laboratory tests, and therefore future work could consider CT scan images.

## Figures and Tables

**Figure 1:** Study framework.

**Figure 2:** System architecture of DMLD prediction model.

**Figure 3:** Classification of data by support vector machine (SVM).

**Figure 4:** Top selected features.

**Figure 5:** Heat map for checking the correlation between selected features.

**Figure 6:** Results of the classifier's performance on the DMLD model.

**Table 1:** Specific liver enzymes with reference ranges.

Liver enzymes	Normal range	Disturbed range	Number of patients with disturbed range
AST	0–0–40	<40	109
ALT	0–37	<37	109

**Table 2:** Data set attributes.

Attribute no.	Attribute	Variable type	Reference range
A1	Creatinine	Real	0.5–1.3
A2	Glucose	Real	70–110
A3	Sodium	Real	135–153
A4	Potassium	Real	3.5–5.3
A5	Calcium	Real	8.8–10.2
A6	Phosphorus	Real	2.7–5
A7	Magnesium	Real	1.5–2.6
A8	Chloride	Real	98–105
A9	Uric acid	Real	3.4–7
A10	Urea	Real	10–50
A11	Albumin	Real	3.4–4.8
A12	Total protein	Real	6.4–8.3
A13	Cholesterol – total	Real	50–200
A14	TG	Real	23–56
A15	ALT	Real	0–37
A16	AST	Real	0–41
A17	Cholesterol – VLDL	Real	10–40
A18	Cholesterol – LDL	Real	50–190
A 19	Cholesterol – HDL	Real	30–70
A 20	LDH	Real	135–225
Class	Liver damage or not	Binary	0 or 1
			0 = healthy liver
			1 = possible liver damage

**Table 3:** Evaluation parameters of different classifiers in the DMLD model.

Predictive models	Accuracy	Precision	Recall
SVM	0.857	0.95	0.95
DT	0.85	0.93	0.93
NB	0.71	0.5	0.5
KNN	0.71	0.5	0.5
ANN	0.7	0.49	0.49

**Table 4:** The impact of different layers on the ANN performance.

Number of layers	Accuracy
1	0.7
3	0.7
4	0.7
5	0.7
10	0.7
15	0.7
20	0.7

## Data Availability

For the privacy of individuals (patients' laboratory results involved in the study), data cannot be made available publicly.
